# An autophagy-related prognostic signature associated with immune microenvironment features of uveal melanoma

**DOI:** 10.1042/BSR20203812

**Published:** 2021-03-19

**Authors:** Zhuotao Zheng, Lingyue Zhang, Zewei Tu, Yan Deng, Xiaolong Yin

**Affiliations:** 1 Department of Pediatric Ophthalmology, The Second Affiliated Hospital of Nanchang University, Nanchang, Jiangxi 330006, P.R. China; 2 Department of Neurosurgery, The Second Affiliated Hospital of Nanchang University, Nanchang, Jiangxi 330006, P.R. China

**Keywords:** autophagy, biomarker, immune microenvironment, prognostic prediction, uveal melanoma

## Abstract

Autophagy is involved in cancer initiation and progression but its role in uveal melanoma (UM) was rarely investigated. Herein, we built an autophagy-related gene (ARG) risk model of UM patients by univariate Cox regression and least absolute shrinkage and selection operator (Lasso) regression model and filtrated out nine prognostic ARGs in The Cancer Genome Atlas (TCGA) cohort. Survival and Receiver Operating Characteristic (ROC) Curve analysis in the TCGA and other four independent UM cohorts (GSE22138, GSE27831, GSE44295 and GSE84976) proved that the ARG-signature possessed robust and steady prognosis predictive ability. We calculated risk scores for patients included in our study and patients with higher risk scores showed worse clinical outcomes. We found the expressions of the nine ARGs were significantly associated with clinical and molecular features (including risk score) and overall survival (OS) of UM patients. Furthermore, we utilized univariate and multivariate Cox regression analyses to determine the independent prognostic ability of the ARG-signature. Functional enrichment analysis showed the ARG-signature was correlated with several immune-related processes and pathways like T-cell activation and T-cell receptor signaling pathway. Gene set enrichment analysis (GSEA) found tumor hallmarks including angiogenesis, IL6-JAK-STAT3-signaling, reactive oxygen species pathway and oxidative phosphorylation were enriched in high-risk UM patients. Finally, infiltrations of several immune cells and immune-related scores were found significantly associated with the ARG-signature. In conclusion, the ARG-signature might be a strong predictor for evaluating the prognosis and immune infiltration of UM patients.

## Introduction

Uveal melanoma (UM) is a type of malignant intraocular cancer derived from melanocytes with high metastasis rate and poor prognosis [1]. Fifty percent patients with UM were found with liver metastases within 10 years from first diagnosis, and the median survival time of patients with metastatic lesions is approx. 5–7 months [2,3]. These data indicated UM is an aggressive tumor with fetal malignancy. However, the methods of cancer biomedical diagnosis and targeted therapy have been developed rapidly in past decades, but the metastasis and death rate of UM did not decline [3]. Nowadays, with the rapid development of biomedical and bioinformatics technologies and methods, universal researches based on cancer expression profiles helped to search cancer diagnostic and therapeutic biomarkers, but similar studies in UM were rare. Therefore, identification of novel and effective prognostic and therapeutic biomarkers remains a priority for UM-tailored therapy.

Autophagy, a cellular programmed-digestion process, has been reported related to several pathological process including malignancy progression. It is a special mechanism for cancer cells to obtain enough energy and nutriment in the hostile conditions of hypoxia, oxidative stress and nutrient starvation [4,5]. In recent years, there emerged numerous autophagy-related cancer researches, and sufficient evidences have revealed that the autophagy process plays a crucial role in the occurrence and progression of various cancers [6–9]. Several autophagy-related genes (ARGs) were revealed associated with the prognosis of cancer patients and were potential biomarkers for predicting the survival time and therapeutic effect for cancer patients [9,10]. However, studies on the role of autophagy in UM are still rare and relative biomarkers or prognostic signatures were hanging for further excavating and developing.

In the present study, we collected five independent UM cohorts (one training cohort and four validation cohorts) and established an autophagy-related prognostic signature by using univariate Cox regression analysis and least absolute shrinkage and selection operator (Lasso) Cox regression in the TCGA training cohort. A risk score was calculated for each patient and by the median value of risk scores we dichotomized patients into low- and high-risk subgroups which showed different overall survival (OS) time and disease-free survival (DFS) time. Besides, functional enrichment analysis between low- and high-risk UM patients showed malignancy-related processes, pathways and signatures are associated with the high-risk patients. Immune microenvironment features, including multiple immune cells, machine-learning based scores, were also investigated for their associations with the ARG-signature in UMs.

## Materials and methods

### Data acquisition

RNA-seq profile and related clinical information of The Cancer Genome Atlas (TCGA) cohort were obtained from the TCGA website (https://portal.gdc.cancer.gov/), and the related RNA expression and clinical information files of the other four cohorts (including GSE22138, GSE27831, GSE44295 and GSE84976) were downloaded from the Gene Expression Omnibus (GEO) repository (https://www.ncbi.nlm.nih.gov/geo/) and previous published researches [11–13]. The baseline information of patients including in current study are summarized in Table 1. The ARGs included in the present study were acquired from the Human Autophagy Database (HADb, http://autophagy.lu/clustering/index.html) [14] and the GO_AUTOPHAGY gene set in the Molecular Signatures Database v6.2 (MSigDB, http://software.broadinstitute.org/gsea/msigdb) [15]. We intersected genes in the five databases and obtained a list of 423 ARGs for further analysis.

**Table 1:** Baseline information of UM patients included in the study

		Training cohort	Validation cohorts			
		TCGA (*n*=80)	GSE22138 (*n*=63)	GSE27831 (*n*=29)	GSE84976 (*n*=28)	GSE39717 (*n*=30)
**OS (year)**						
	Range (Median)	0.01–7.12 (2.08)	0.01–9.91 (2.61)	/	1.17–13.00 (5.50)	0.00–7.48 (1.85)
**DFS (year)**						
	Range (Median)	/	/	1.23–5.51 (3.29)	/	/
**Age (years)**						
	≤60	40 (50%)	28 (44.44%)	/	12 (42.86%)	11 (36.67%)
	>60	40 (50%)	35 (55.56%)	/	16 (57.14%)	19 (63.33%)
**Gender**						
	Male	45 (56.25%)	39 (61.90%)	/	/	23 (76.67%)
	Female	35 (43.75%)	24 (38.10%)	/	/	7 (23.33%)
**M stage**						
	Yes	3 (37.50%)	35 (55.56%)	11 (37.93%)	14 (50.00%)	8 (26.67%)
	No	73 (91.25%)	28 (44.44%)	18 (62.07%)	14 (50.00%)	22 (73.33%)
	NA	4 (5.00%)	0 (0.00%)	0 (0.00%)	0 (0.00%)	0 (0.00%)
**N stage**						
	Yes	0 (0.00%)	/	/	/	/
	No	76 (95.00%)	/	/	/	/
	NA	4 (5.00%)	/	/	/	/
**T stage**						
	T2	4 (5.00%)	/	/	/	/
	T3	36 (45.00%)	/	/	/	/
	T4	38 (47.50%)	/	/	/	/
	NA	2 (2.50%)	/	/	/	/
**Histology**						
	Epithelioid	13 (16.25%)	21 (33.33%)	/	/	/
	Mixed	37 (46.25%)	23 (36.51)	/	/	/
	Spindle	30 (37.50%)	0 (0.00%)	/	/	/
	NA	0 (0.00%)	19 (30.16%)	/	/	/
**Thickness (mm)**						
	≤10	37 (46.25%)	10 (15.87%)	/	/	/
	>10	43 (53.75%)	53 (84.13%)	/	/	/
	NA	0 (0.00%)	0 (0.00%)	/	/	/
**Chr 6p gain**						
	Yes	23 (28.75%)	/	/	/	/
	No	57 (71.25%)	/	/	/	/
	NA	0 (0)	/	/	/	/
**Chr 8q gain**						
	Yes	32 (40.00%)	/	/	/	/
	No	48 (60.00%)	/	/	/	/
	NA	0 (0)	/	/	/	/
**Chr1 loss**						
	Yes	9 (11.25%)	/	/	/	/
	No	71 (88.75%)	/	/	/	/
	NA	0 (0)	/	/	/	/
**Chr3 loss**						
	Yes	31 (38.75%)	37 (58.73%)	/	14 (50.00%)	/
	No	49 (61.25%)	18 (28.57%)	/	14 (50.00%)	/
	NA	0 (0)	8 (12.70%)	/	/	/

### Data processing

For the TCGA RNA-seq cohort, The Fragments Per Kilobase of transcript per Million (FPKM) values were transformed to Transcripts Per Kilobase Million (TPM) values according to an algorithm acquired in published researches [16,17]. For the microarray data in the GSE22138, GSE27831, GSE44295 and GSE84976 cohort, background adjustments and quantile normalization were performed on the microarray raw data using a robust multiarray averaging method (RAM) with the R packages ‘affy’ [18] and ‘simpleaffy’ [19]. The TPM and RAM expression values in each cohort were utilized in following data analysis.

### Construction of the ARG-signature

By taking the TCGA cohort as training cohort, we performed univariate Cox regression analysis to the 423 ARGs based on the survival information in the TCGA cohorts and we screened out 133 OS-related ARGs (*P*<0.05) including 39 protective ARGs (HR < 1) and 94 risky ARGs (HR > 1). These OS-related ARGs were used to further construct the prognostic signature by Lasso Cox regression analysis. Finally, a 9-ARG signature was established and a risk score calculating formula, based on the related expression value and coefficients of the nine ARGs, was developed. The formula developed was as following:

$$Risk\;\;score\;=\;\sum_{i=1}^{n}Coef_{i}\;\times \;x_{i}$$

in which the $Coef_{i}$ is the coefficient of each ARGs, and $x_{i}$ is the TPM value or RMA value of each ARG in each cohort.

Based on the formula above, risk scores were calculated for each patients and divided UM patients into low- and high-risk subgroups by the median risk score in each cohort.

### Functional enrichment analysis

Genes whose expressions were in significant differential levels between low- and high-risk UM patients with |log2 (fold change)| > 1 and *P*-value <0.05 were defined as differential expression genes (DEGs) in the present study. We used the R package ‘limma’ [20] to perform differential expression analysis in the TCGA cohort and we obtained 2365 DEGs. Then the R package ‘clusterProfiler’ [21] was used to perform Gene Ontology (GO) and Kyoto Encyclopedia of Genes and Genomes (KEGG) pathway analysis based on the 2365 DEGs. The software ‘GSEA’ (version 4.0.1) was the main platform to identify significant cancer hallmarks between low- and high-risk UM patients with the standards of Normalized Enrichment Score (NES) ≥ 1, Normalized *P*-value (Norm *P*) <0.05 and False Discovery Rate (FDR) < 0.25.

### Immune cells infiltration and immune-related scores calculation

Based on the TPM expression values of UM patients in the TCGA cohort, the 22 immune cells infiltration proportions of each UM patients were calculated using ‘CIBERSORT’ R package. The ESTIMATE score, immune score, stromal score and tumor purity values of UM patients in the TCGA dataset were obtained from the website of PanCanAtlas Publications (https://gdc.cancer.gov/about-data/publications/panimmune).

### Statistical methods

Two-sided log-rank test was applied to contrast the OS/DFS between different risk subgroups or expression levels of ARGs of UM patients in survival curves, visualized by R package ‘survival’. To evaluate the OS/DFS predictive power of the ARG-signature, receiver operating characteristic (ROC) curves were plotted by R package ‘timeROC’ [22] and area under curve (AUC) was calculated as the main quantized parameter. Based on the clinical and survival information, univariate and multivariate Cox regression were the vital analytical methods to decide the independent prognostic role of the ARG-signature. The analysis method of correlations between risk scores and immune-related scores was Pearson correlation analysis. Statistical analysis contained in our study were implemented based on the R programming language (version 3.6.3, https://www.r-project.org/).

## Results

### Development of the ARG-signature in UM patients

The workflow of the development of the risk signature is shown as Figure 1. To develop an ARG-signature which could be applied to all the patients in these five cohorts, we first examined the detection statuses of the 531 ARGs in each cohort. By taking the intersection of the detected ARGs, we finally obtained a list of shared 423 ARGs in all the cohorts.

**Figure 1:** Flow chart of the construction and validation of the ARG-signature

Then univariate Cox regression analysis showed that 133 of the 423 ARGs were associated with the OS of UM patients in the TCGA cohort (*P*<0.05), of which 39 ARGs were protective genes (HR < 1) and 94 ARGs were risky genes (HR > 1). Lasso Cox regression model was subsequently applied to the 133 OS-related ARGs to establish a prognostic model for the UM patients in the TCGA cohort. We successfully developed a prognostic signature based on nine ARGs (Figure 2A,B). The coefficients of the nine ARGs were visualized from high to low in the Figure 2C, and univariate Cox regression analysis of the nine ARGs were summarized in Table 2.

**Figure 2:** Construction of the ARG-signature (**A,B**) Lasso regression was performed to calculate the minimum criteria and coefficients for constructing the ARG-signature. (**C**) The histogram exhibits the coefficients of the nine ARGs. (**D**) The survival curves indicate that UM patients with higher risk scores were significantly associated with worse OS time. (**E**) The survival distribution plot showing that patients with higher risk scores are associated with shorter OS. (**F**) ROC curves showing the 1-, 3-, and 5-year OS predictive efficiency of the ARG-signature. (**G**) The heatmap showed the correlations between the expression levels of the 9 ARGs and clinical and molecular features (including the ARG-signature) of UM patients in the TCGA cohort.

**Table 2:** Univariate Cox regression analysis of the nine ARGs in the TCGA cohort

ARGs	HR	HR.95L	HR.95H	*P*-value	Coefficient
**TUSC1**	2.1716	1.5322	3.0778	<0.0001	−0.0606
**LMCD1**	0.6813	0.5515	0.8418	0.0004	−0.0480
**GABARAPL1**	1.0242	1.0125	1.0361	<0.0001	−0.0411
**PRKCD**	0.8149	0.7370	0.9010	0.0001	−0.0319
**DLC1**	1.6332	1.3017	2.0491	<0.0001	−0.0146
**FKBP1A**	1.9597	1.4198	2.7050	<0.0001	0.0035
**ITGA6**	0.1594	0.0571	0.4447	0.0005	0.0930
**BNIP1**	0.8626	0.7972	0.9333	0.0002	0.1349
**IKBKE**	0.6954	0.5867	0.8243	<0.0001	0.1870

To confirm the prognostic predictive value of the ARG-signature, 80 UM patients were separate into 40 low- and 40 high-risk patients by the median risk score in the TCGA cohort. The Kaplan–Meier curves (survival analysis) revealed that low-risk UM subgroup have higher survival rate and longer survival time compared with the high-risk subgroup (Figure 2D). And the patients’ distributions plot depicted that high-risk UM patients showed shorter OS time compared with low-risk patients (Figure 2E). Besides, the ROC analysis indicated that the risk score possessed a very high AUC value for predicting the 1/3/5-year OS of UM patients (Figure 2F, 1/3/5-year AUC = 0.907/0.953/1.000), which means the ARG-signature have a pretty robust predictive accuracy.

Furthermore, associations between the 9-gene expression levels and clinical and molecular features (including risk score) were investigated. UM patients were in order with the risk score increasing and patients with higher risk were associated with lower DLC1, GABARAPL1, LMCD1, PRKCD, TUSC1 expressions, higher BNIP1, ITGA6 IKBKE and FKBP1A expressions, more Chr3/Chr8q loss, less Chr6p loss and higher tumor thickness, diagnostic age and clinical stage (Figure 2G).

### Validation of the ARG-signature in external cohorts

Generally, a well-performed prognostic signature needs more validations in other retrievable cohorts. Prognostic validation analysis was used to verify the prognostic predictive stability of the ARG-signature. In the GSE44295 cohort, 57 UM patients were divided into low- and high-risk UM groups by the median risk score and survival analysis showed that high-risk UMs were associated with lower OS rate and shorter OS time (Figure 3A), patients’ distributions of OS time and status also proved this result (Figure 3B). And ROC curves revealed the risk score remained a high level of prognostic predictive ability in the GSE44295 cohort (Figure 3C, 1/3/5 AUC = 0.833/0.745/0.731). Similar results were also found in the GSE84976 (*n*=28) and GSE22138 (*n*=63) UM cohorts (Figure 3D–I), it showed that the ARG-signature could commendably distinguish between low- and high-risk UMs with distinct OS time.

**Figure 3:** Prognostic predictive ability of the ARG-signature Survival curves, survival distribution plot and ROC curves showed the ARG-signature could accurately predict the OS or DFS of patients and in the GSE84976 (**A**–**C**), GSE22138 (**D**–**F**), GSE39717(**G**–**I**) and GSE27831 (**J–L**).

Furthermore, the GSE27831 cohort (*n*=29) was used to examined whether the ARG-signature could predict the DFS of UM patients. Like the results above, DFS analysis and patients’ distributions of DFS time indicated that the high-risk UM patients have a lower DFS rate and shorter DFS time (Figure 3J,K). And ROC curves demonstrated that the ARG-signature could well forecast the 3/5-year DFS of UM patients (Figure 3L).

### The prognostic value of the nine ARGs

Survival analysis was used to test the relationship between the OS and ARGs’ expression in the TCGA cohort, UM patients were divided into low- and high-expression of each genes to compare survival difference between two subgroups. UM patients with high expression levels of IKBKE, BNIP1, ITGA6 and FKBP1A showed worse clinical outcomes which means they might be risky ARGs in UM (Figure 4A–D). And high expression levels of DLC1, PRKCD, GABARAPL1, LMCD1 and TUSC1 were associated with better clinical outcomes of UM patients, the five ARGs could be potential protective genes in UM (Figure 4E–I). The results of survival analysis were consistent with the univariate Cox regression results (Table 2).

**Figure 4:** Prognostic roles of the nine ARGs (**A–D**) Survival analysis represented high expressions of IKBKE (A), BNIP1 (B), ITGA6 (C) and FKBP1A (D) were correlated with worse clinical outcomes of UM patients. (**E–I**) Survival analysis represented high expressions of DLC1 (E), PRKCD (F), GABARAPL1 (G), LMCD1 (H) and TUSC1 (I) were correlated with better clinical outcomes of UM patients.

### Independent prognostic ability of the ARG-signature stratification

Univariate and multivariate Cox regression were implemented to examine the independent prognostic role of the ARG-signature in the TCGA cohort. We concluded clinically common factors like gender, age, stage, T and M statuses (N status was excluded due to there exists 76 N0 UMs and 4 Nx UMs) in the univariate Cox regression analysis. The results of univariate Cox regression showed higher age (HR: 1.046, 95% CI: 1.008–1.085, *P*=0.019), clinical stage (HR: 2.902, 95% CI: 1.149–7.330, *P*=0.024), M status (HR: 49.280, 95% CI: 4.434-547.731, *P*=0.002), T status (HR: 2.439, 95% CI: 1.032–5.763, *P*=0.042) and risk stratification (HR: 3.857, 95% CI: 2.595–5.732, *P*<0.001) were significantly associated with prognosis of UM patients, and gender (HR: 1.542, 95% CI: 0.651–3.652, *P*=0.325) was not a prognostic predictor (Figure 5A).

**Figure 5:** Prognostic role of the ARG-signature (**A,B**) Univariate Cox regression and multivariate analyses showed the ARG-signature was an independent prognostic risk factor of UM patients in the TCGA cohort. (**C,D**) Survival analysis indicated that the ARG-signature could divide UM patients into low- and high-risk subgroups independent of chemotherapy (C) of radiotherapy (D). (**E,F**) Principal component analysis (PCA) showed that low-risk and high-risk UM patients could be distinguished based on all genes’ expression or ARGs’ expression.

Factors with statistical significance in the univariate Cox regression were included in the multivariate Cox regression analysis and results showed that the M stage (HR: 24.99, 95% CI: 1.074–581.502, *P*=0.045) and the risk stratification (HR: 4.243, 95% CI: 2.501–7.196, *P*<0.001) possessed independent prognostic roles (Figure 5B).

We noticed that half of UM patients in the TCGA received radiotherapy and the other half of UM patients were under chemotherapy. To excluded the effects of different therapy methods, we applied survival analysis in UM patients with different therapy and results indicated that UM patients with higher risk scores have worse clinical outcomes no matter what treatment they received (Figure 5C,D).

Principle component analysis (PCA) showed UM patients were in distinct directions based on all detected genes or 531 ARGs profiles in the TCGA cohort (top three principle components were analyzed), which indicated that UM patients with different risk stratification harbored different gene expression status and autophagy status (Figure 5E,F).

### Functional enrichment analysis

To investigate the inner molecular distinctions between low- and high-risk UM patients, DEGs between low- and high-risk patients were analyzed in the TCGA cohort. Differential expression analysis was first performed between low- and high-risk subgroups of UM patients in the TCGA cohort and 2369 DEGs were identified.

In order to understand the main functional processes and pathways of the 2369 DEGs, we implemented GO and KEGG pathway to identify the dominating functions of them. Results of GO analysis revealed that functional enrichments of these DEGs included T-cell activation, lymphocyte activation, leukocyte activation and differentiation (biological process, BP), plasma membrane protein complex, extracellular matrix, collagen-containing extracellular matrix (cellular component, CC), receptor regulator activity, channel activity, passive transmembrane transporter activity (molecular function, MF) and so on (Figure 6A). KEGG pathway analysis indicated that cytokine–cytokine receptor interaction, cell adhesion molecules (CAMs), antigen processing and presentation, Th1 and Th2 cell differentiation, natural killer cell-mediated cytotoxicity, Th17 cell differentiation, T cell receptor signaling pathway and NF-κB signaling pathway were significantly differentially enriched between low- and high-risk UM patients (Figure 6B).

**Figure 6:** Functional enrichment analysis between low- and high-risk UM patients (**A**) Gene ontology BP (GO-BP) analysis of DEGs between low- and high-risk UM patients in the TCGA cohort. (**B**) KEGG pathway analysis of DEGs between low- and high-risk UM patients in the TCGA cohort. (**C**) Gene set enrichment analysis (GSEA) of hallmarks enriched in high-risk UM patients in the TCGA cohort.

Tumor hallmarks were also investigated between low- and high-risk UM patients in the TCGA cohort by using gene set enrichment analysis (GSEA) method. We identified four tumor hallmarks including Angiogenesis, IL6-JAK-STAT3 signaling, Reactive oxygen species pathway and Oxidative phosphorylation were prominently enriched in high-risk UM patients (Figure 6C).

### ARG-signature related immune microenvironment features

In light of the results of functional enrichment analysis, we speculated that the ARG-signature was associated with the immune characterization of UM. The landscape of 22 immune cell infiltration proportions were shown in Figure 7A. The violin plot was used to visualize the differences of immune cell infiltration between low- and high-risk UM samples (Figure 7B). Results showed that B cell naive, T cells CD4 memory resting, Monocytes, Mast cells resting were significantly infiltrating in low-risk UM samples and T cells CD8, T cells CD4 memory activated and T cells follicular helper were more infiltrating in high-risk UM patients.

**Figure 7:** Immune cell infiltration analysis of UM samples (**A**) Proportion of 22 immune cells calculated by CIBERSORT algorithm of each UM samples were shown between low- and high-risk UM patients. (**B**) Statistical significance of the proportion of 22 immune cells between low- and high-risk UM patients. (**C–F**) Pearson correlation analysis showed the risk score was significantly associated with the ESTIMATEScore (C), TumorPurity (D), Immune score (E) and Stromal score (F) calculated using machine-learning methods. *P<0.05, **P<0.01, ***P<0.001.

Immune microenvironment-related scores, including ESTIMATE score, Tumor Purity, Immune score and Stromal score, were calculated for each patients using related algorithm. These immune microenvironment related scores were used to performed Pearson correlation analysis with the risk score to confirm the correlation between the ARG-signature and immune microenvironment status. Results showed that the risk score was positively associated with the ESTIMATE score (R = 0.43, *P*=6.1⁁-5), Immune score (R = 0.46, *P*=2⁁-5) and Stromal score (R = 0.31, *P*=0.0048) and negatively associated with the Tumor Purity (R = −0.43, *P*=8.1⁁-5). These data demonstrated that UM patients with higher risk scores were infiltrated with more immune and stromal cells.

## Discussion

Along with booming evolution of biotechnological and bioinformatics science, genomic analysis had been widely applied to search cancer biomarkers or develop diagnostic and prognostic models [23]. However, few associated studies focused on prognostic prediction model development of UM patients. In current research, we combined univariate Cox regression model and Lasso Cox regression model to screen OS-related ARGs and developed a prognostic ARG-signature to distinguish patients with distinct clinical outcomes. Furthermore, unlike previous prognostic signature development researches [24], the ARG-signature was successfully validated in other four external independent UM cohorts, it is the greatest strength of our study and it proved the robustness and stableness of our ARG-signature. Nevertheless, the main limitation of our study was the number of patients included might not be enough compared with counterpart researches in other cancer types, although we have tried to search UM cohorts for validation.

ROC curve analysis was the main method to judge the prognostic prediction accuracy of the ARG-signature in our study, and we noticed that the AUC value of the 5-year OS prediction in the TCGA cohort and the 5-year DFS prediction in the GSE27831 cohort was 1.000, which might raise some concerns about the accuracy of our risk model. These results might be contributed by the reason that only three patients and one patient lived longer than 5 year in the TCGA and GSE27831 cohorts, respectively. On the contrary, there were 18, 9 and 17 UM patient lived longer than 5 years in GSE22138, GSE44295 and GSE84976 cohorts, respectively.

In current study, we totally identified nine prognostic ARGs and found high expressions of IKBKE, BNIP1, ITGA6, FKBP1A and low expressions of DLC1, PRKCD, GABARAPL1, LMCD1 and TUSC1 were associated with worse prognosis of UM patients. Inhibitor of nuclear factor κ B kinase subunit ϵ (IKBKE) had been discovered as an oncogene and is overexpressed in over 30% of breast carcinomas samples and cell lines [25]. It was reported that BNIP1 could restrain cervical cancer cell proliferation, migration and invasion by inhibit mTOR signaling pathway, although it seemed to be a risky factor in UM patients [26]. Integrin subunit α 6 (ITGA6), a member of the integrin α chain family of proteins, is an efficient early-detection biomarker and prognostic factor for colorectal cancer patients [27]. FKBP1A belongs to immunophilin protein family and mediate the immunosuppressive and antitumor effects of rapamycin [28]. DLC-1 is a Rho GTPase-activating protein (RhoGAP), could facilitate melanoma cell invasion and metastasis by cooperating transcription factor FOXK1 to promote MMP9 expression [29] and enhancing colorectal cancer metastasis by the epithelial-to-mesenchymal transition [30]. The protein kinase C δ (PRKCD) is a member of the protein kinase C family of serine- and threonine-specific protein kinases and it is involving in manipulating tumor repopulation while receiving radiotherapy [31]. It had been reported that lower GABARAPL1 expression is correlated with poor prognosis of hepatocellular carcinoma and lymph node-positive breast cancer patients [32,33], which might indicate that GABARAPL1 is a negative regulator of cancer progression. LIM and cysteine-rich domains 1 (LMCD1) had been found acting as an activator E2F1 transcription factor in human cells [34] but its role in cancers were rarely investigated. TUSC1 tumor suppressor candidate 1 (TUSC1) is a putative tumor suppressor gene and could restrain lung cancer and glioblastoma cells growth *in vitro* [35,36]. Few researches focused on the roles of the nine ARGs in UM and we thought our work could help to throw light on the roles of them.

In conclusion, totally 257 UM patients in five independent cohorts were included and used to develop and validate a prognostic predictive signature for UM patients. The ARG-signature showed a powerful predictive ability to the clinical outcomes in both training cohort and four external validation cohorts. Meanwhile, nine novel prognostic ARGs were identified associated with the clinical outcomes of UM patients and might provide some clues for further researches. Besides, UM patients with higher risk scores showed higher immune cell infiltration levels and tumor hallmarks enrichments.

## Data Availability

The data analyzed in the present study can be accessed the TCGA (http://cancergenome.nih.gov/) and GEO (https://www.ncbi.nlm.nih.gov/geo/) websites.

## Abbreviations

ARG: autophagy-related gene
AUC: area under curve
DEG: differential expression gene
DFS: disease-free survival
GEO: Gene Expression Omnibus
GSEA: gene set enrichment analysis
HR: harzard ratio
KEGG: Kyoto Encyclopedia of Genes and Genomes
Lasso: least absolute shrinkage and selection operator
OS: overall survival
RAM: robust multiarray averaging method
ROC: receiver operating characteristic
TCGA: The Cancer Genome Atlas
TPM: Transcripts Per Kilobase Million
UM: uveal melanoma
95%CI: 95% confidence interval
